# RIPK3 interactions with MLKL and CaMKII mediate oligodendrocytes death in the developing brain

**DOI:** 10.1038/cddis.2017.54

**Published:** 2017-02-23

**Authors:** Yi Qu, Jun Tang, Huiqing Wang, Shiping Li, Fengyan Zhao, Li Zhang, Q Richard Lu, Dezhi Mu

**Affiliations:** 1 Department of Pediatrics, West China Second University Hospital, Sichuan University, Chengdu 610041, China; 2 Key Laboratory of Birth Defects and Related Diseases of Women and Children (Sichuan University), Ministry of Education, Chengdu 610041, China; 3 Department of Pediatrics, Division of Experimental Hematology and Cancer Biology, Cincinnati Children's Hospital Medical Center, Cincinnati 45229, OH, USA; 4 Department of Pediatrics, University of California, San Francisco, CA 94143, USA

## Abstract

Oligodendrocyte progenitor cells (OPCs) death is a key contributor to cerebral white matter injury (WMI) in the developing brain. A previous study by our group indicated that receptor-interacting proteins (RIPs) are crucial in mediating necroptosis in developing neurons. However, whether this mechanism is involved in OPCs death is unclear. We aimed to explore the mechanisms of RIP-mediated oligodendrocytes (OLs) death in the developing brain. Oligodendrocytes necroptosis was induced by oxygen-glucose deprivation plus caspase inhibitor zVAD treatment (OGD/zVAD) *in vitro*. Western blotting and immunofluorescence were used to detect RIPK1, RIPK3, mixed lineage kinase domain-like protein (MLKL), and Ca^2+^ and calmodulin-dependent protein kinase II*δ* (CaMKII*δ*). Immunoprecipitation was used to assess the interactions between RIPK3 and RIPK1, MLKL, and CaMKII*δ*. Necrostatin-1 was used to disturb the RIPK3–RIPK1 interaction, and siRNA was used to inhibit RIPK3 or MLKL expression. Oligodendrocytes death was examined using PI staining, EM, and cell membrane leakage assays. *In vivo*, brain damage in neonatal rats was induced by hypoxia–ischemia (HI). This was followed by an examination of myelin development. We found that OGD/zVAD treatment upregulates the expression of RIPK3 and the interaction of RIPK3 with RIPK1, MLKL, and CaMKII*δ*. Inhibition of the RIPK3-MLKL or RIPK3-CaMKII*δ* interaction attenuates OLs death induced by OGD/zVAD. These protective mechanisms involve the translocation of MLKL to the OLs membrane, and the phosphorylation of CaMKII*δ*. However, inhibition of the RIPK3–RIPK1 interaction did not protect OLs death induced by OGD/zVAD. *In vivo* studies indicated that the disrupted development of myelin was attenuated after the inhibition of RIPK3-MLKL or RIPK3-CaMKII*δ* interaction. Taken together, our data indicate that RIPK3 is a key factor in protection against OLs death and abnormal myelin development via its interaction with MLKL and CaMKII*δ* after HI. This suggests that RIPK3 may be a potential target for the treatment of WMI in neonates.

With rapid advances in neonatal intensive care, the survival rate of premature infants has been significantly improved. However, many survivors of preterm birth have severe sequelae, such as cerebral palsy.^1^ At present, the most common type of brain injury in preterm neonates is white matter injury (WMI), wherein the loss and impaired maturation of oligodendrocytes (OLs) result in neuropsychiatric problems.^2^ Preterm birth is associated with maternal inflammation, perinatal infections, and disrupted oxygen supply, which may affect the cerebral microenvironment by causing activation of microglia, astrogliosis, excitotoxicity, and oxidative stress. This intricate interplay of events leads to OLs death and disrupted maturation of OLs, which ultimately result in myelination failure in the developing white matter.^3^ OLs development is strictly regulated during the perinatal period. In the first stage of OLs development, neural stem cells differentiate into oligodendrocyte progenitor cells (OPCs), which express a panel of membrane-bound markers, such as A2B5 and the proteoglycan neural/glial antigen 2 (NG2). As differentiation progresses, they develop into premyelinating oligodendrocytes (pre-OLs), which can be identified with an array of markers, including O4. Fully mature OLs enwrap axons with myelin in a process called myelination. At this stage, cells express specific myelin proteins, such as myelin basic protein (MBP).^4^ Neonates born between 24 and 30 weeks of gestation are at high risk for WMI, as vulnerable OPCs and pre-OLs are the predominating cells of the OLs lineage in the brain at this gestational age.^5^ The death of OPCs results in the depletion of the mature OLs pool and subsequent abnormal development of myelin in the cerebral white matter, which in turn leads to impaired neurological function.^6^ Therefore, exploring the mechanisms mediating OPCs death is crucial. Research in this area will help to find new strategies for the prevention and treatment of white matter diseases.

Apoptosis has generally been considered to be the predominant mechanism of regulated cell death. In recent years, however, another important type of cell death, necroptosis, has been described as an alternative cell death pathway.^7^ Receptor-interacting proteins (RIPs), especially RIPK1 and RIPK3, have been shown to be crucial factors in the initiation of cell necroptosis.^8, 9^ They form the backbone of a large necrosome, which is an essential platform for the recruitment of other components and stimulates the downstream execution of necroptosis.^10^ Mixed lineage kinase domain-like protein (MLKL) is prominent among the recruited components.^11^ The RIPK3-MLKL interaction leads to the phosphorylation and oligomerization of MLKL, which in turn leads to the disruption of cell membrane integrity.^11, 12^

Recently, Ca^2+^ and calmodulin-dependent protein kinase II*δ* (CaMKII*δ*) was identified as a new RIPK3 substrate. CaMKII is a serine/threonine protein kinase with four isoforms (*α*, *β*, *δ*, and *γ*) that are encoded by different genes displaying distinct but overlapping expression patterns.^13^ Each isoform contains an N-terminal kinase domain, a regulatory Ca^2+^/calmodulin (Ca^2+^/CaM)-binding region, and a C-terminal association domain. The four different CaMKII isoforms possess similar catalytic and regulatory properties.^14^ CaMKII is activated by two distinct processes when it binds Ca^2+^/CaM. One is the phosphorylation of threonine-287 (Thr287), and the other is oxidation of methionine-281/282.^15^ Phosphorylation is a critical feature of CaMKII function, as it allows the kinase to translate transient changes in calcium concentration into sustained enzyme activity.^16^ Recent research indicates that at least two pathways are involved in the RIPK3-mediated activation of CaMKII*δ*. The two pathways are the direct phosphorylation of CaMKII Thr287 by RIPK3 and its indirect reactive oxygen species (ROS)-mediated oxidation. Both of these activation pathways contribute to RIPK3-induced myocardial necroptosis.^17^ Furthermore, dissipation of the mitochondrial membrane potential (ΔΨm) has been shown to be an essential downstream event in RIPK3-activated CaMKII*δ* signaling.^17^

A previous study by our group has revealed that both RIPK1 and RIPK3 are crucial in mediating necroptosis in neurons subjected to hypoxia–ischemia (HI).^18^ Therefore, we hypothesized that RIP-mediated necroptosis is also involved in OLs death. We used cell and animal models of HI to demonstrate that RIPK3, but not RIPK1, is indispensable in mediating HI-induced OLs death. We found that the interactions of RIPK3 with MLKL and CaMKII*δ* are involved in HI-induced OLs death, which suggests that RIPK3 might be a potential target in attenuating OLs death in the developing brain.

## Results

### Necroptosis is induced in OPCs with oxygen-glucose deprivation plus caspase inhibitor zVAD insult (OGD/zVAD)

We investigated whether necroptotic death occurs when OPCs are submitted to OGD, an *in vitro* model of HI. Meanwhile, zVAD, a broad-spectrum caspase inhibitor, was used to facilitate cell death from apoptosis to necroptosis. As the result, OGD or OGD/zVAD insult induced membrane permeability that is observable as propidium iodide (PI)-positive staining 24 h after OGD (Figure 1a). On electron microscopy (EM), a morphological pattern that had characteristics of necroptosis was observed 24 h after OGD, including both the accumulation of cytoplasmic vacuoles, as seen in classical necrosis, and the compaction of chromatin into a few, discrete, large clumps, as seen in classical apoptosis (Figure 1b). We also found OPCs membrane leakage was induced by both OGD and OGD/zVAD. Twenty-four hours after OGD insult, cell death reached ~62% in OGD OPCs and 68% in OGD/zVAD OPCs (Figure 1c).

### OGD/zVAD upregulates RIPK3 expression, and RIPK3-MLKL and RIPK3-CaMKII*δ* interactions without affecting RIPK1 expression

As the RIPK1-RIPK3-MLKL and RIPK3-CaMKII*δ* interactions are reported to be involved in the induction of necroptosis,^17, 19^ we investigated the RIPK1-RIPK3-MLKL and RIPK3-CaMKII*δ* interactions in OPCs subjected to OGD/zVAD insult. Western blotting showed that RIPK3 protein was upregulated 6 h and remained high until 48 h after OGD, immunofluorescent staining demonstrated increased RIPK3 expression in OGD/zVAD group compared with the controls 12 h after OGD, whereas RIPK1, MLKL, and CaMKII*δ* expression levels were not obviously changed (Figures 2a and b). Immunoprecipitation showed increases in the RIPK3–RIPK1, RIPK3-MLKL, and RIPK3-CaMKII*δ* interactions in the OGD/zVAD group 12 h after OGD (Figure 2c).

### Downregulation of the RIPK3-MLKL or the RIPK3-CaMKII*δ* interaction attenuated OPCs death after OGD/zVAD

As the RIPK3–RIPK1, RIPK3-MLKL, and RIPK3-CaMKII*δ* interactions were significantly upregulated in OPCs subjected to OGD/zVAD insult, we examined the roles of these interactions in regulating OPCs death. When Necrostatin-1 (Nec-1), the RIPK1 inhibitor, was used, the RIPK3–RIPK1 interaction was attenuated, whereas the RIPK3-MLKL and RIPK3-CaMKII*δ* interactions were unaffected 12 h after OGD (Figure 3a). Nec-1 treatment did not affect OPCs death in the OGD/zVAD group 24 h after OGD (Figure 3a). In contrast, RIPK3 siRNA treatment significantly reduced RIPK3 expression, the RIPK3-MLKL interaction, and the RIPK3-CaMKII*δ* interaction 12 h after OGD, and OPCs death 24 h after OGD (Figure 3b).

### MLKL oligomerization was enhanced in the membrane fraction of OPCs after OGD/zVAD insult

The RIPK3-MLKL interaction has been reported to induce MLKL oligomerization and membrane translocation, thus mediating necroptosis in some cell types.^12, 18^ We therefore analyzed MLKL in the membrane and non-membrane fractions of OPCs using SDS-PAGE under non-reducing conditions. As shown in Figure 4, MLKL existed in the non-membrane fractions largely as monomers (~50 kDa) under normal culture conditions but formed an oligomer larger than 250 kDa in membrane fractions 12 h after OGD when OPCs were subjected to OGD/zVAD. Furthermore, we found that RIPK3 inhibition via siRNA attenuated the oligomerization of MLKL in OPCs membrane fractions in the OGD/zVAD group 12 h after OGD (Figure 4).

### Calcium influx was increased in OPCs cultured in glucose-free medium

Calcium influx into cells has recently been reported to be a downstream effector of MLKL during the induction of necroptosis.^12^ To detect calcium influx during necroptosis, OPCs were loaded with the calcium indicator Fluo-3/AM. We found that Fluo-3/AM fluorescence was markedly increased in OPCs after glucose was removed from the culture medium. Furthermore, knocking down RIPK3 in OPCs attenuated glucose deprivation-induced calcium influx, suggesting that RIPK3 is required for calcium influx in OPCs (Figures 5a–c).

### CaMKII*δ* was activated through phosphorylation but not oxidation in OPCs after OGD/zVAD insult

RIPK3 activates CaMKII*δ* via direct phosphorylation (p287-CaMKII) or indirect oxidation by evoking ROS in cardiomyocytes.^17^ Therefore, we investigated whether CaMKII*δ* activation is increased in OPCs following OGD/zVAD insult. We found that phospho-Thr287 CaMKII*δ* levels were increased in OPCs in the OGD/zVAD group 12 and 24 h after OGD, whereas total CaMKII*δ* levels were not affected. Furthermore, RIPK3 inhibition via siRNA decreased phospho-Thr287 CaMKII*δ* levels (Figure 6a). In contrast, CaMKII*δ* oxidation was not enhanced in OPCs 12 or 24 h after OGD (Figure 6b), and ROS production was not increased 12 h after the OGD/zVAD insult (Figure 6c). In the presence of butylated hydroxyanisole (BHA) or N-acetylcysteine (NAC), which are two widely used ROS scavengers, OPCs in the OGD/zVAD group also underwent cell death 24 h after OGD (Figure 6d). This suggests that ROS is dispensable in the process of OPCs death after OGD/zVAD insult.

### ΔΨm collapsed after OGD/zVAD insult in OPCs

CaMKII*δ* activation can trigger the opening of the mitochondrial permeability transition pore, resulting in the depolarization of the ΔΨm and necroptosis in cardiomyocytes.^17^ We therefore examined ΔΨm in OPCs after OGD/zVAD insult. ΔΨm was measured using the JC-1 fluorescence ratio, which is the average optical density ratio of red/green. A low ratio represents a dissipation of ΔΨm. Our results indicate that OGD/zVAD leads to the dissipation of ΔΨm in OPCs after 24 h, whereas RIPK3 inhibition via siRNA attenuates the dissipation of ΔΨm and enhances OPCs survival 24 h after OGD (Figure 7a). When KN-93, which is a selective inhibitor of CaMKII, was used, CaMKII*δ* phosphorylation was inhibited 12 h after OGD, and the dissipation of ΔΨm was attenuated. We also observed enhanced survival of OPCs in the OGD/zVAD group 24 h after OGD (Figure 7b).

### Inhibition of the RIPK3-MLKL interaction or the RIPK3-CaMKII*δ* interaction attenuated the disruption of myelin development in neonatal rats subjected to HI

A well-described model of subcortical WMI was generated using P6 rats.^20, 21^ RIPK3 siRNA significantly inhibited the expression of RIPK3 12 and 24 h after HI and interrupted the RIPK3-MLKL and RIPK3-CaMKII*δ* interactions 24 h after HI. In addition, MLKL siRNA significantly inhibited the expression of MLKL 12 and 24 h after HI and interrupted the RIPK3-MLKL interaction 24 h after HI. KN-93 significantly inhibited the phosphorylation of CaMKII*δ* 24 h after HI (Figure 8a). We found that the numbers of OPCs (NG2-positive cells) were significantly decreased in the ipsilateral hemisphere 24 h after HI. We also observed a marked decrease in MBP expression at P14. The inhibition of the RIPK3-MLKL interaction or the RIPK3-CaMKII*δ* interaction via siRNA or the inactivation of CaMKII*δ* with KN-93 attenuated OPCs depletion 24 h after HI and MBP loss at P14. However, there were no significant differences in MBP levels between rats in the HI and sham groups at P21 (Figure 8b). Nevertheless, the ultra-structure of myelin under EM was obviously different between the HI and sham groups at P21. In sham rats, myelin was well-developed and had a compact structure. On the other hand, in the HI-exposed rats, myelin exhibited obvious stratification and fragmentation, which indicate disrupted myelin development (Figure 8c). Disturbance of the RIPK3-MLKL interaction or the RIPK3-CaMKII*δ* interaction and inhibition of CaMKII*δ* phosphorylation partly attenuated the disruption of myelin development (Figures 8b and c).

## Discussion

In the present study, we found that necroptotic cell death occurs when OLs are subjected to OGD, which is used as an *in vitro* model of HI. OGD/zVAD insult upregulates RIPK3 and increases the RIPK3–RIPK1, RIPK3-MLKL, and RIPK3-CaMKII*δ* interactions. Furthermore, the inhibition of the RIPK3-MLKL or RIPK3-CaMKII*δ* interactions attenuates OLs death induced by OGD/zVAD. The mechanism underlying this effect involves the translocation of oligomerized MLKL to the OLs membrane and the phosphorylation of CaMKII*δ* after OGD/zVAD insult. However, inhibition of the RIPK3–RIPK1 interaction does not affect OLs death induced by OGD/zVAD. Experiments in neonatal rats subjected to HI further indicated that disrupting either the RIPK3-MLKL interaction or the RIPK3-CaMKII*δ* interaction counters the abnormal development of myelin. This is the first study to suggest that RIPK3 plays a key role in mediating HI-induced OLs death in the developing brain. The mechanisms underlying this effect are summarized in Figure 9.

Recent studies have indicated that non-apoptotic cell death is present in many pathological processes. The classical study on necroptosis by Junying Yuan found that neuronal necroptosis may occur under ischemic conditions in the absence of exogenous caspase inhibitors.^7^ The authors of that study speculated that this phenomenon might result from the development of an apoptosis-nonpermissive environment upon ischemic injury due to insufficient cellular energy supplies. They also proposed that necroptosis may function as the primary cell death mechanism in some populations of cells. Here we found that both OGD and OGD/zVAD treatments induced the same PI-positive staining and morphological pattern of necroptosis (Figure 1), suggesting that necroptosis might be the primary cell death mechanism for OPCs under OGD circumstances. This finding is in line with those of previous studies showing that OGD-induced OLs death occurs in a non-apoptotic manner.^22, 23^ Although most of the OPCs undergo necroptosis after OGD insult without zVAD, to ensure that the largest number of OPCs is available for the study of the mechanisms regulating necroptosis, we used zVAD to ensure that the cells died in a necroptotic manner. The use of zVAD to establish an *in vitro* necroptotic cell model has been widely used in the field of necroptosis research,^7^ and is proven to be useful in mechanistic studies. Unfortunately, there have been no standard bio-markers for necroptosis until now, especially *in vivo*.^24^ The relevance of the cell death with classical necroptosis-modulating molecules, such as RIPK1 and RIPK3, might provide evidence of the occurrence of necroptosis.

Nec-1 has been reported to abolish the RIPK1-RIPK3 interaction, inhibit RIPK3 phosphorylation, and attenuate necroptosis.^8^ However, in the current study, Nec-1 did not attenuate HI-induced OPCs death despite inhibiting the RIPK3–RIPK1 interaction. Previous studies have reported that in addition to the RIPK1-RIPK3 interaction, RIPK3–RIPK3 dimerization can induce necroptosis. RIPK3 dimerization leads to RIPK3 intramolecular autophosphorylation, which is sufficient for the recruitment of downstream effectors.^25^ Another study indicates that overexpression of RIPK3 reduces the requirement for RIPK1 in necroptosis initiation.^26^ Based on these findings, we deduced that the overexpression of RIPK3 in OPCs subjected to HI might lead to a massive increase in the formation of RIPK3–RIPK3 dimers, which are sufficient for the activation of downstream effectors of necroptosis. Our findings further indicate that RIPK1 might be dispensable as a mediator of cell death under some circumstances.

The mechanism downstream of MLKL in necroptosis is very complicated, and is tissue- and cell-type specific. Recently, Wang *et al.*^27^ reported that phosphorylated MLKL can form oligomers and move from the cytoplasm to the cell membrane, where it binds to phosphatidylinositol lipids and cardiolipin, inserts deeply into the membrane bilayer, and directly disrupts membrane integrity, finally resulting in cell death. Here, we find that MLKL forms tetramers and translocates from the cytoplasm to the OPCs membrane after OGD/zVAD insult. This may in turn induce OPCs death by directly disrupting membrane integrity.

Besides MLKL, the present study also revealed that CaMKII*δ* is crucial in mediating OL death after OGD/zVAD insult. We found that CaMKII*δ* is activated through phosphorylation but not oxidation in OPCs after OGD/zVAD insult. This process was found to be indispensable in mediating OPCs death. When KN-93 was used, CaMKII*δ* phosphorylation was inhibited and the dissipation of ΔΨm was largely attenuated. This led to enhanced survival of OPCs after OGD/zVAD insult. KN-93 has been known to be a selective inhibitor of CaMKII that attenuates CaMKII phosphorylation by competitively blocking Ca^2+^/CaM binding to the kinase. The powerful effects of KN-93 on reversing the pro-necrotic role of RIPK3 suggest that phosphorylation of CaMKII*δ* by RIPK3 occurs in a Ca^2+^/CaM-dependent manner.

Our *in vivo* studies provide a kinetic vision of OLs damage. We detected OPCs (NG2-positive) 24 h after HI and mature OLs (MBP-positive) 14 and 21 days after HI. This allowed us to observe the time course of OLs damage following HI. We found that the numbers of OPCs were significantly decreased 24 h after HI. We also observed a marked decrease in MBP expression at P14. Although MBP levels were not significantly different at P21, the ultra-structure of myelin under EM was obviously different between the HI and sham groups at P21. This suggests that OLs depletion during the earlier period of HI insult results in lasting disruption of myelin development. This indicates that strategies for the attenuation of OLs death are pivotal in protection against WMI in neonates. Therefore, RIPK3, which is the crucial molecule mediating OLs death in the developing brain, might serve as a potential target for the prevention and treatment of WMI in neonates.

## Materials and methods

### Primary culture of OPCs

All animal protocols were approved by the Sichuan University Committee on Animal Research and complied with the ARRIVE guidelines. Primary rat OPCs were prepared from the cerebral hemispheres of Sprague-Dawley rats on postnatal day 1 (P1) using a shaking method^28^ with modifications, as previously described.^29^ Purified OLs were cultured for 7 days in a serum-free basal-defined medium (BDM): DMEM (Invitrogen, Carlsbad, CA, USA), 10 ng/ml human recombinant platelet-derived growth factor (Peprotech, Rocky Hill, NJ, USA), 10 ng/ml human recombinant basic fibroblast growth factor (Peprotech), 0.1% bovine serum albumin (Sigma, St. Louis, MO, USA), 10 nM hydrocortisone (Sigma), 200 *μ*M L-cystine (Sigma), 50 *μ*g/ml insulin (Sigma), 30 nM sodium selenite (Sigma), 10 nM d-biotin (Sigma), and 50 *μ*g/ml human apo-transferrin (Sigma). The expression of stage-specific OL lineage markers, such as A2B5 (progenitors), O4 (later-stage precursors), O1 (immature OL), and MBP (mature OL) was monitored routinely by immunostaining. A representative OPCs culture had the following composition: 95% A2B5+, 90% O4+, 4% O1+, and 1% MBP+. Besides, all cultures contained less than 2% of glial fibrillary acidic protein-positive astrocytes and non-detectable CD11+ microglia.

### Oxygen-glucose deprivation

To test the effects of Nec-1 (20 *μ*M, Sigma), BHA (100–200 *μ*M, Sigma), NAC (0.05–10 mM, Sigma), and KN-93 (10 *μ*M, Sigma), cells were pretreated with each of the reagents at the mentioned concentrations together with zVAD (20 *μ*M, Sigma) for 1 h, followed by OGD insult. Control groups were treated with vehicle (DMSO, Sigma) together with zVAD for 1 h, followed by OGD insult. This dosing schedule of drugs was selected based on the results of previous reports.^12, 30, 31^

To initiate OGD, cultures were switched to BDM medium that lacked glucose (Invitrogen) and were transferred to a chamber filled with 94% N_2_/5% CO_2_/1% O_2_ at 37 °C. Following OGD for 2.5 h, d-glucose was added back to the cultures to a final concentration of 25 mM, and the cultures were returned to an air/5% CO2 incubator at 37 °C. Cell death was assessed by PI staining, EM, and a cell membrane leakage assay. Molecular changes were examined by western blotting, immunofluorescent staining, and immunoprecipitation at the indicated time points after OGD insult.

### RNA interference

Small interfering RNA duplexes (siRNA) targeting *RIPK3* (ID246240) (si-RIPK3, Ribobio, Guangzhou, China) or nonspecific sequences (Scrambled) (si-Scr, Ribobio) without modification were synthesized. Ten nmol of siRNA was transfected into the cells. The same concentration of the nonspecific sequence was used as the scrambled control. Cells were cultured for 24 h and subjected to OGD, as above.

### Transmission EM

Cells or brain tissues were fixed in phosphate-buffered saline (PBS) containing 2% paraformaldehyde/2% glutaraldehyde for 60 min. After washing in the same buffer, cells were gently scraped off and centrifuged. Cells or brain tissues were then post-fixed with 1% OsO_4_, 0.8% potassium ferricyanide, and 5 mM CaCl_2_ in 0.1 M cacodylate buffer, dehydrated in acetone and embedded in Epox 812 (EMS, Baton Rouge, LA, USA) overnight at 60 °C. Ultrathin sections (90 nm) were stained with uranyl acetate and lead citrate and observed under an H-600IV transmission electron microscope (Hitachi, Tokyo, Japan).

### Detection of cell death using PI staining

PI (1 mg/ml, Sigma) and Hoechst 33258 (10 mg/ml, Sigma) were added to media and incubated with the cells for 5 min. Photographs were randomly taken from three individual 200 × fields per well to quantify PI-positive cells. There were six wells per experimental condition. PI-positive cells were expressed as a percentage of Hoechst-positive cells.

### Cell membrane leakage assay

A cell membrane leakage assay was performed using the CytoTox-Glo Cytotoxicity Assay Kit according to the manufacturer's instructions (Promega, Madison, WI, USA). Luminescence was recorded with a microplate reader (Thermo Varioskan Flash, Waltham, MA, USA).

### Immunofluorescent staining

Cells on coverslips were blocked (1 × PBS, 2% normal goat serum, and 0.1% Triton X-100) for 1 h and incubated overnight at 4 °C with the following primary antibodies: anti-RIPK1 (1:400; Abcam, Burlingame, CA, USA), anti-RIPK3 (1:400, Abcam), anti-MLKL (1:400, Abcam), and anti-CaMKII*δ* (1:100; GeneTex, Irvine, CA, USA). Cells were washed three times with 0.1 M PBS and then incubated with Cy3-labeled secondary antibody (1:400; Beyotime, Shanghai, China) for 1 h at room temperature. The cells were then photographed under a fluorescent microscope (Leica, Microsystems, Wetzlar, Germany) with an excitation wavelength of 550 nm and an emission wavelength of 570 nm.

### Crude cell membrane fraction

Cells (2.5 × 10^6^ cells) were detached from the culture plates with a non-enzymatic solution consisting of HBSS (Sigma) with 1 mM EDTA (Sigma) and washed twice with PBS (Sigma). Cells were resuspended in 1 ml of the fractionation buffer (250 mM sucrose, 20 mM HEPES at pH 7.4, 10 mM KCl, 1.5 mM MgCl_2_, 1 mM EDTA, and 1 mM EGTA) and placed on ice for 10 min. Cells were disrupted by freezing with liquid nitrogen for 5 min and then thawing on ice, repeating this sequence three times. The lysates were passed through a 25G needle (BD Biosciences, San Jose, CA, USA) 10 times. Nuclei and unbroken cells were removed by centrifugation at 750 × *g* for 5 min. The supernatant was collected and centrifuged again at 10 000 × *g* for 5 min. The supernatant was then centrifuged at 100 000 × *g* in an Optima TLX Ultracentrifuge (Beckman Coulter, Brea, CA, USA) for 1 h at 4 °C. The supernatants containing cytosolic proteins were concentrated using an acetone precipitation method. The pellets containing membrane proteins were washed with the fractionation buffer and were re-centrifuged at 100 000 × *g* for 45 min. The pellets were collected and lysed in M2 buffer (20 mM Tris, pH 7, 0.5% NP40, 250 mM NaCl, 3 mM EDTA, 3 mM EGTA, 2 mM DTT, 0.5 mM phenylmethylsulphonyl fluoride, 20 mM glycerol phosphate, 1 mM sodium vanadate, and 1 *μ*g/ml leupeptin). For reducing gel analysis, normal SDS-PAGE was performed as described below. For non-reducing gel analysis, cells were lysed in M2 buffer without DTT and separated by SDS-PAGE without mercaptoethanol.

### Western blotting

Cells were lysed in ice-cold lysis buffer (10 mM Tris-HCl, pH 7.8, 100 mM NaCl, 10 mM EDTA, 0.5% Nonidet P-40, and 0.5% sodium deoxycholate) supplemented with protease and phosphatase inhibitors. Homogenates were maintained in ice for 30 min and centrifuged at 15 000 × *g* for 10 min at 4 °C, and the supernatant was recovered. Protein concentration was determined by BCA protein assay kit (Life, New York, NY, USA). Proteins were resolved in SDS-PAGE (10% polyacrylamide), transferred to PVDF membrane, and incubated with primary antibodies. The reactions were followed by incubation with peroxidase labeled secondary antibodies (Life). Primary antibodies used were: anti-RIPK1 (1:800, Abcam), anti-RIPK3 (1:800; Abcam), anti-MLKL (1:1000, Abcam), anti-*β*-actin (1:5000, Abcam), anti-Na+-K+-ATPase (1:400; Santa Cruz, Santa Cruz, CA, USA), anti-CaMKII*δ* (1:800, GeneTex), anti-p-CaMKII (1:800, Thermo), and anti-ox-CaMKII (1:600; Millipore, Bedford, MA, USA). CaMKII activation was assessed by measuring phosphorylation and oxidation levels.

### Immunoprecipitation

Cells were homogenized in cold lysis buffer, and the lysed samples were precleared by adding resuspended Protein A/G PLUS-Agarose (Santa Cruz). Samples were incubated at 4 °C for 30 min and centrifuged for 8 min at 2500 × *g*, and the pellet was discarded. Protein (250 *μ*g) was combined with an anti-RIPK3 antibody (2 *μ*g, Abcam) and incubated overnight, gently mixing at 4 °C. Immobilized protein A (Life) 100 *μ*l was added to the antigen–antibody complex and gently mixed at room temperature for 2 h. To remove any unbound protein, the samples were washed 4 times with 0.5 ml of immunoprecipitation buffer (Life) and centrifuged for 3 min at 2500 × *g*. The supernatant was discarded after each wash. The pellet was washed with 0.5 ml distilled H_2_O, centrifuged for 3 min at 2500 × *g*, and the supernatant discarded. The beads were resuspended in 50 *μ*l of 2 × treatment buffer, boiled for 5 min, and then centrifuged at 14 000 × *g* for 5 s. The supernatant (20 *μ*l per lane) was loaded onto a gel for SDS-PAGE. Blots were incubated overnight at 4 °C with anti-RIPK1, anti-MLKL, or anti-CaMKII*δ*, and then exposed to the corresponding secondary antibody and developed with enhanced chemiluminescence. The same amount of irrelevant IgG (Santa Cruz) was used as the nonspecific binding control.

### Intracellular calcium concentration measurements using laser confocal scanning microscopy

Intracellular calcium concentration [Ca^2+^]i was measured using the Fluo-3/AM staining method as described by Chen.^31^ A solution of 0.1% Pluronic F127 was added to a Fluo-3-AM/DMSO solution (500 *μ*M) to prevent aggregation of Fluo-3/AM in HBSS and to help uptake by the cells. The Fluo-3-AM solution was diluted with HBSS to prepare 5 *μ*M Fluo-3-AM working solution. Cells were incubated with Fluo-3/AM for 30 min in the dark at room temperature. The dye-loaded cells were gently washed three times with Ca^2+^-free HEPES-buffered saline. The cells were kept in normal or glucose-free medium for a further 1 h in the dark. Fluorescence was then detected using a confocal laser scanning microscope (LSM 700, Carl Zeiss, Jena, Germany). In brief, fluorescence was elicited by excitation with a 488-nm argon laser line at an approximate rate of two frames per second. The fluorescence intensities were detected at a wavelength of 528 nm. Fluorescence images were scanned and stored as a time series. Emitted fluorescence was collected using a 20 × objective. The data obtained from the first and second scans were considered the basal data for [Ca^2+^]i, and the maximum fluorescence intensity in each cell was considered to be the peak for [Ca^2+^]i. Fifteen individual cells in the regions of interest were randomly selected in each group for determination of the average fluorescence intensities.

### Measurement of ROS

We used 5-(and-6)-chloromethyl-2, 7-dichlorodihydrofluorescein diacetate acetyl ester (DCF, Invitrogen) to assess ROS production in cultured cells. After washing with PBS, cells were incubated with 10 *μ*M DCF for 30 min, allowed to recover for 15 min in full growth medium, and washed again with PBS. Fluorescence was measured at 483 nm excitation and 520 nm emission using a laser scanning system (LSM 700, Carl Zeiss) and analyzed using ImageJ software (NIH, Bethesda, MD, USA).

### Assessment of ΔΨm

To measure the ΔΨm, JC-1 (Molecular Probes, Eugene, OR, USA), which is a sensitive fluorescent probe for ΔΨm, was used according to the manufacturer's protocol. Cells were washed with PBS and incubated with 2 *μ*g/ml JC-1 at 37°C for 30 min. After removing JC-1 and washing the cells with PBS, images were captured using a fluorescence microscope (Nikon, TiE, Japan) with both red and green channels. Ten nonadjacent fields in each group were selected randomly for statistical analysis. IPP 6.0 software was used to measure the average red and green fluorescent intensity in each group. The ΔΨm is represented by the JC-1 fluorescence ratio. The JC-1 fluorescence ratio was calculated as the average red/green fluorescent intensity ratio.

### Myelin development in neonatal rats

WMI was induced in postnatal day 6 (P6) rats using unilateral carotid ligation followed by hypoxia (6% O_2_ for 1 h), as described previously.^20, 21^ Rats were anesthetized using ether, and the proximal internal carotid artery was isolated from the sympathetic chain, clamped, and cauterized. The neck wound was closed, and the animals were allowed to recover for 1 h. The rats were then placed in a sealed chamber infused with nitrogen to a level of 6% O_2_. After 1 h of recovery, the rats were returned to their dam. Sham control rats were subjected to isolation and stringing of vessels without occlusion and subsequent ischemia.

For *in vivo* gene delivery, rat pups immediately after right common carotid artery ligation were given a single intracerebroventricular injection of methyl and cholesterol modified small interfering RNA duplexes (siRNA) targeting *RIPK3* (ID246240) (si-RIPK3, Ribobio), *MLKL* (ID690743) (si-MLKL, Ribobio), or nonspecific sequences (Scrambled) (si-Scr, Ribobio), followed by hypoxia treatment as described above. For each rat, 1 nmol siRNA plus 0.5 nmol transfection control (Ribobio) were complexed and injected into the lateral ventricle using a Hamilton syringe with a 26-gauge needle. Cy3 was used to monitor success of transfection. To inhibit the activation of CaMKII, KN-93 (10 *μ*mol/kg) was injected intraperitoneally into rat pups daily for 3 days before HI insult. At the indicated time points after the HI insult, the ipsilateral brain tissue were collected and used for western blotting and immunoprecipitation, according to the methods described above. NG2-positive cells were immunostained using an anti-NG2 antibody (1:300, Abcam).

Oligodendrocyte maturation was evaluated by immunostaining with antibodies against the specific OL marker MBP on alternating serial 10-*μ*m-thick coronal sections, as detailed previously.^20, 21^ Sections were blocked and incubated overnight with an anti-MBP monoclonal antibody (1:100, Millipore). Sections were rinsed and then incubated with the appropriate secondary antibody (Pierce Biotechnology, Rockford, IL, USA) for 1 h at room temperature. MBP expression was assessed in three regions (medial, middle, and lateral) along the corpus callosum in each hemisphere of each section and graded using a modified five-point scoring system:^21^ 0, immunohistochemical staining hardly visible; 1, faint staining of the corpus callosum with rarefaction of the periventricular WM and loss of fibrillar features; 2, thinning of the corpus callosum with broken fibrillar processes; 3, few cortical processes or supracallosal fibers without cortical processes; and 4, thick corpus callosum with dense and extended cortical processes. The scores for each region were summed up to obtain a total score (range, 0–12) for each ipsilateral hemisphere. Four coronal sections, two at the level of the striatum (0.26 mm and 0.92 mm posterior to the bregma) and another two at the level of the dorsal hippocampus (3.14 mm and 4.16 mm posterior to the bregma), according to a rat brain atlas,^32^ were analyzed and averaged for each brain. Two independent observers, blind to the treatment conditions, measured the MBP scores. Furthermore, the ultra-structure of myelin was assessed using transmission EM, as described above.

### Statistical analysis

Data are presented as means±S.E.M. from three independent experiments. Student's *t*-tests were used when comparing two groups. Analyses of variance and Fisher's *post hoc* tests were used when comparing more than two groups. Values of *P*<0.05 were considered significant.

## Figures and Tables

**Figure 1:** Necroptosis is induced in OPCs following OGD/zVAD insult. (**a**) Representative images and quantification of PI-positive OPCs treated with OGD or OGD/zVAD. Photographs were randomly taken from three individual 200 × fields per well 24 h after OGD. There were six wells per experimental condition. The numbers of PI-positive cells are expressed as percentages of Hoechst-positive cells. Data are presented as means ±S.E.M. from three independent experiments (Scale bar=20 *μ*m) (*P<0.05, comparing the OGD or OGD/zVAD group with the sham group). (**b**) Observation of OPCs 24 h after OGD using electron microscopy revealed a morphological pattern with features of necroptosis. An accumulation of cytoplasmic vacuoles was observed, as seen in classical necrosis, whereas nuclei underwent compaction of chromatin into a few discrete, large clumps, similar to classical apoptosis. This was inconsistent with the formation of numerous smaller, irregular chromatin clumps observed during classical necrosis (Scale bar=2 *μ*m). Arrows indicate large clumps in the nucleus. (**c**) OPCs death was determined kinetically by measuring released protease activity in culture medium. The data are represented as means±S.E.M. from three independent experiments. *N*=6 for each group in each experiment (*P<0.05, comparing the OGD or OGD/zVAD group with the sham group)

**Figure 2:** OGD/zVAD upregulates RIPK3 expression, and the RIPK3-MLKL and RIPK3-CaMKII*δ* interactions without affecting RIPK1 protein expression. (**a**) Western blotting was used to determine protein expression levels. The ratios of the levels of the indicated proteins to that of *β*-actin were calculated and normalized to the value in the sham control group. We found that RIPK3 protein was upregulated 6 h after OGD and remained high until 48 h after OGD, whereas the expression levels of RIPK1, CaMKII*δ*, and MLKL were not affected by the OGD insult. (**b**) Immunofluorescence staining 12 h after OGD indicated increased RIPK3 expression after the OGD/zVAD insult compared with the sham controls, whereas RIPK1, CaMKII*δ*, and MLKL expression levels were not obviously changed. Arrows indicate representative positive staining cells, and insets show these cells at higher magnification (scale bar=40 *μ*m). (**c**) Immunoprecipitation was carried out 12 h after OGD to assess the interactions between RIPK3 and RIPK1, MLKL, or CaMKII*δ*. We found increases in the RIPK3–RIPK1, RIPK3-MLKL, and RIPK3-CaMKII*δ* interactions after OGD/zVAD insult. Data are presented as means±S.E.M. from three independent experiments. *N*=6 for each group in each experiment (*P*<0.05, compared with the sham control). S: sham; O/z: OGD/zVAD

**Figure 3:** Downregulation of the RIPK3-MLKL interaction or the RIPK3-CaMKII*δ* interaction attenuates OPCs death after OGD/zVAD. (**a**) Immunoprecipitation 12 h after OGD shows that the RIPK3–RIPK1 interaction was decreased after Nec-1 treatment, whereas the RIPK3-MLKL and RIPK3-CaMKII*δ* interactions were not decreased. Cell death, as determined by measuring released protease activity in the culture medium 24 h after OGD, was not affected after Nec-1 treatment. Data are presented as means±S.E.M. from three independent experiments. *N*=6 for each group in each experiment. S: sham; O/z: OGD/zVAD; N: Nec-1; Ni: Nec-1 inhibitor. (**b**) Western blotting indicates that RIPK3 siRNA treatment significantly reduced RIPK3 expression 12 h after OGD. Immunoprecipitation assays showed that the RIPK3-MLKL and RIPK3-CaMKII*δ* interactions were decreased 12 h after OGD following the inhibition of RIPK3 via RIPK3 siRNA treatment. Cell death, as determined by measuring the released protease activity in the culture medium, was significantly decreased 24 h after OGD following RIPK3 inhibition. Data are presented as means±S.E.M. from three independent experiments. *N*=6 for each group in each experiment (*P*<0.05, comparing the siRNA group with the OGD/zVAD group). S: sham; O/z: OGD/zVAD; Si: RIPK3 siRNA; Sc: RIPK3 siRNA scramble

**Figure 4:** MLKL oligomerization is enhanced in the membrane fraction of the OPCs after OGD/zVAD insult. OPCs were subjected to OGD/zVAD. Total, non-membrane, and membrane fractions were then resolved on either reducing or non-reducing gels and analyzed by western blotting. MLKL was largely in the non-membrane fraction as monomers (~50 kDa) under normal culture conditions, but formed an oligomer larger than 250 kDa in the membrane fraction in OPCs 12 h after OGD/zVAD. siRNA-mediated RIPK3 inhibition attenuated the oligomerization of MLKL in the OPCs membrane fraction in the OGD/zVAD group 12 h after OGD. The absence of Na^+^-K^+^-ATPase in the non-membrane fraction indicated that there was no cross-contamination between the non-membrane and membrane fractions. T, total cell lysate; NM, non-membrane fraction; M, membrane fraction; S: sham; O/z: OGD/zVAD; Si: RIPK3 siRNA; Sc: RIPK3 siRNA scramble

**Figure 5:** Calcium influx is increased in OPCs cultured in glucose-free medium. (**a**) Intracellular calcium concentration ([Ca^2+^]i) in OPCs was measured using the Ca^2+^ indicator Fluo-3 under laser confocal scanning microscopy. Fluo-3/AM fluorescence was markedly increased in OPCs after culture in glucose-free medium. Furthermore, RIPK3 inhibition via siRNA attenuated the glucose deprivation-induced calcium influx (scale bar=40 *μ*m). (**b**) The mean fluorescence intensity curve for [Ca^2+^]i in each group with different treatments. Data are presented as means±S.E.M. from three independent experiments. *N*=6 for each group in each experiment. (**c**) Basal and peak fluorescence intensity for [Ca^2+^]i in each group. Data are presented as means±S.E.M. from three independent experiments. *N*=6 for each group in each experiment (*P*<0.05, comparing the siRNA group with the OGD/zVAD group). S, sham; GD, glucose deprivation; Si, RIPK3 siRNA; Sc, RIPK3 siRNA scramble

**Figure 6:** CaMKII*δ* is activated via phosphorylation, but not oxidation, in OPCs after OGD/zVAD insult. (**a**) Representative western blotting images and averaged data indicating phosphorylated and total CaMKII*δ* levels in OPCs. Phospho-Thr287 CaMKII*δ* levels were increased in OPCs in the OGD/zVAD group 12 and 24 h after OGD, whereas total CaMKII*δ* was not affected. Furthermore, RIPK3 inhibition via siRNA decreased phospho-Thr287 CaMKII*δ* levels 12 and 24 h after OGD. Data are presented as means ±S.E.M. from three independent experiments. *N*=6 for each group in each experiment (*P*<0.05, comparing the siRNA group with the OGD/zVAD group). S: sham; O/z: OGD/zVAD; Si: RIPK3 siRNA; Sc: RIPK3 siRNA scramble. (**b**) Representative western blotting images and averaged data for oxidation of CaMKII*δ* (ox-CaMKII) at M281/282. In the sham control group, CaMKII*δ* oxidation is very weak. OGD/zVAD insult did not enhance CaMKII*δ* oxidation in OPCs 12 or 24 h after OGD. Data are presented as means±S.E.M of three independent experiments. *N*=6 for each group in each experiment. S: sham; O/z: OGD/zVAD; Si: RIPK3 siRNA; Sc: RIPK3 siRNA scramble. (**c**) Representative photomicrographs of ROS production as assessed using DCF staining (green). 4',6-diamidino-2-phenylindole (DAPI) was used as the counterstain in order to highlight the nucleus (blue). ROS production was not increased in OPCs in the OGD/zVAD group 12 h after OGD (scale bar=20 *μ*m). S: sham; O/z: OGD/zVAD; Si: RIPK3 siRNA; Sc: RIPK3 siRNA scramble. (**d**) OPCs were treated with vehicle, BHA, or NAC at the indicated concentrations together with zVAD 1 h before the OGD insult. Cell death was assessed by measuring the released protease activity in the culture medium. In the presence of these ROS scavengers, OPCs also underwent cell death 24 h after OGD. Data are presented as means±S.E.M. from three independent experiments. *N*=6 for each group in each experiment. S, sham; O/z, OGD/zVAD; V, vehicle

**Figure 7:** ΔΨm collapses after OGD/zVAD insult in OPCs. (**a**) Representative photomicrographs of JC-1 staining and quantification of the JC-1 fluorescence ratio. The JC-1 fluorescence ratio was calculated using the average red/green optical density ratio. A low ratio represents a dissipation of ΔΨm. OGD/zVAD led to dissipation of ΔΨm in OPCs 24 h after OGD. RIPK3 inhibition via siRNA attenuated the dissipation of ΔΨm and enhanced OPCs survival 24 h after OGD. Data are presented as means ±S.E.M. from three independent experiments. *N*=6 for each group in each experiment (scale bar=40 *μ*m) (*P*<0.05, comparing the siRNA group with the OGD/zVAD group). S: sham; O/z: OGD/zVAD; Si: RIPK3 siRNA; Sc: RIPK3 siRNA scramble. (**b**) KN-93 inhibits CaMKII*δ* phosphorylation in OPCs in the OGD/zVAD group 12 h after OGD, attenuates the dissipation of ΔΨm 24 h after OGD, and enhances OPCs survival 24 h after OGD. Data are presented as means±S.E.M. from three independent experiments. *N*=6 for each group in each experiment. (Scale bar=40 *μ*m) (*P*<0.05, comparing the KN-93 group with the OGD/zVAD group). S, sham; O/z, OGD/zVAD; KN-93, CaMKII inhibitor; KN-92, negative control for KN-93

**Figure 8:** Inhibition of the RIPK3-MLKL interaction or the RIPK3-CaMKII*δ* interaction attenuates the disruption of myelin development in neonatal rats subjected to HI insult. (**a**) Western blotting and immunoprecipitation assays on the ipsilateral brain tissue indicate that RIPK3 siRNA significantly reduces RIPK3 expression 12 and 24 h after HI, and that the interactions of RIPK3 with MLKL and CaMKII*δ* are decreased 24 h after HI. MLKL siRNA significantly reduced MLKL expression 12 and 24 h after HI and the RIPK3-MLKL interaction 24 h after HI. KN-93 significantly inhibited CaMKII*δ* phosphorylation 24 h after HI. Data are presented as means ±S.E.M. from three independent experiments. *N*=6 for each group in each experiment (*P*<0.05, comparing the Si group with the Sc group; or comparing the KN-93 group with the negative control KN-92 group). (**b**) Representative images of immunostaining for NG2 and MBP in the corpus callosum of the ipsilateral hemisphere and quantification of the MBP score. The MBP score was assessed in three regions (medial, middle, and lateral) along the corpus callosum in each section. Four sections per brain were analyzed. Data are presented as means±S.E.M. from three independent experiments. *N*=6 for each group in each experiment. The number of OPCs (NG2-positive cells) was significantly decreased in the ipsilateral hemisphere 24 h after HI. There was also a marked decrease in MBP expression at P14. However, at P21, MBP levels were not significantly different between HI and sham rats. Inhibition of RIPK3 and MLKL via siRNA, or inactivation of CaMKII with KN-93, attenuated OPCs depletion 24 h after HI and increased MBP levels at P14 (scale bar=40 *μ*m) (*P*<0.05, comparing the Si group with the Sc group; or comparing the KN-93 group with the KN-92 group). (**c**) Representative transmission electron microscopy images of the ultra-structure of myelin at P21. Myelin was well-developed with a compact structure in sham rats, whereas in the HI rats, myelin exhibited obvious stratification and fragmentation. Inhibition of RIPK3 and MLKL via siRNA, or inactivation of CaMKII with KN-93, partly attenuated the disruption to myelin development (scale bar=2 *μ*m). S: sham; HI: hypoxia–ischemia; Si: RIPK3 or MLKL siRNA; Sc: RIPK3 or MLKL siRNA scramble; KN-93: CaMKII inhibitor; KN-92: negative control for KN-93

**Figure 9:** Summary of the mechanisms underlying RIPK3-mediated OPCs death induced by HI
